The article "Circular RNA hsa_circ_0002360 Promotes Proliferation and Invasion and Inhibits Oxidative Stress in Gastric Cancer by Sponging miR-629-3p and Regulating the PDLIM4 Expression" was retracted in 2023. Reasons: unreliable results or conclusions; lack of ethics approval or compliance; concerns about the data; concerns about the peer review.

# Circular RNA hsa_circ_0002360 Promotes Proliferation and Invasion and Inhibits Oxidative Stress in Gastric Cancer by Sponging miR-629-3p and Regulating the PDLIM4 Expression

**DOI:** 10.1155/2022/2775433

**Published:** 2022-08-09

**Authors:** Zhengyuan Yu, Jing Lan, Wei Li, Li Jin, Feng Qi, Chen Yu, Hao Zhu

**Affiliations:** ^1^Department of Medical Oncology, The First Affiliated Hospital of Soochow University, No. 188, Shizi Street, Gusu District, Suzhou 215006 Jiangsu, China; ^2^Department of General Surgery, The First Affiliated Hospital of Soochow University, No. 188, Shizi Street, Gusu District, Suzhou 215006 Jiangsu, China; ^3^Department of Radiotherapy, Sichuan Cancer Hospital & Institute, Sichuan Cancer Center, School of Medicine, University of Electronic Science and Technology of China, 55# Renmin South Road, 610041 Chengdu, Sichuan, China; ^4^Department of Pharmacy, The Fourth Affiliated Hospital of Nantong University, Yancheng City No. 1 Peoples' Hospital, Yancheng, 224006 Jiangsu, China; ^5^Department of Integrated TCM & Western Medicine, Jiangsu Cancer Hospital & Jiangsu Institute of Cancer Research & The Affiliated Cancer Hospital of Nanjing Medical University, Nanjing, China; ^6^Department of Traditional Chinese Medicine, The First Affiliated Hospital of Soochow University, No. 188, Shizi Street, Gusu District, Suzhou 215006 Jiangsu, China

## Abstract

Many studies have found that circRNA hsa_0002360 (circ0002360) plays an important role in cancer onset and progression. However, its role in gastric cancer (GC) remains uncertain. Circ0002360 was found to be upregulated in GC cells using QRT-PCR. Furthermore, miR-629-3p, a target miRNA of circ0002360, was the most suppressed miRNA following circ0002360 overexpression. RNA immunoprecipitation (RIP), dual-luciferase reporter analyses, clone formation, transwell, DCFH-DA, and ELISA assays demonstrated that circ0002360-targeted miR-629-3p promotes cell proliferation and migration while inhibiting oxidative stress. GC-related mRNA microarrays from the GEO and TCGA databases, including GSE103236, GSE79973, GSE33429, GSE22804, GSE84437, and TCGA-STAD datasets, were used to find hub biomarkers between normal and gastric cancer samples. WGCNA and uni-Cox analysis were used to identify 27 survival-related risk genes, which were then used to build a risk model for prognosis prediction. Following that, all patients from the GSE84437 and TCGA-STAD datasets with 27 survival-related genes and enough data on survival status and time were randomly assigned to train (*n* = 433) and test (*n* = 375) cohorts. Furthermore, ROC and Kaplan-Meier (KM) analyses were used to validate the risk model for both cohorts. randomForest analysis indicated that PDLIM4 was the target gene of miR-629-3p, whose level was increased by circ0002360 but reversed by miR-629-3p mimics. Finally, this study confirmed that circ0002360 sponged miR-629-3p and then upregulated PDLIM4 expression. As a result, circ0002360 may be a useful marker for predicting GC prognosis and an anti-GC treatment target.

The article "Circular RNA hsa_circ_0002360 Promotes Proliferation and Invasion and Inhibits Oxidative Stress in Gastric Cancer by Sponging miR-629-3p and Regulating the PDLIM4 Expression" was retracted in 2023. Reasons: unreliable results or conclusions; lack of ethics approval or compliance; concerns about the data; concerns about the peer review.

## 1. Introduction

Gastric cancer (GC) is a malignant gastrointestinal (GI) tumor that ranks 5th and 3rd in the world in terms of morbidity and factors contributing to cancer-associated mortality [1]. The data show that GC causes increasing morbidity and mortality in Asian countries, especially in China, Japan, and South Korea [2]. Due to the uneven regional distribution of medical resources in our country, the prevalence of early GC screening remains low. Many GC cases are in an advanced tumor progression stage at the time of initial diagnosis, making surgical treatment difficult, with a high metastasis rate and poor prognosis [3–5]. Currently, early symptom occurrence and pathologic transformation of GC are considered to be a pathologic process with diverse stages, multiple influencing factors, and slow progression [6, 7]. Changes in gene expression, mutations, and epigenetics are also strongly associated with the progression of GC [8]. Because of increased social and environmental pressures and dietary changes, the incidence of GC has risen in recent years, and the aggressive, differentiated, and bulky tumors of young and middle-aged patients with GC impose a significant mental and physical burden [9, 10]. As a result, it is particularly vital to explore molecular diagnostic markers, prognostic factors, and personalized therapeutic markers that can guide clinical diagnosis.

Circular RNAs (circRNAs) are single-stranded RNAs found in eukaryotes that are specifically expressed in specific tissue types and developmental stages. CircRNAs can be produced by back-splicing precursor mRNA (pre-mRNA) transcripts, resulting in a covalently-closed ring architecture with no 3′ poly-A tail or 5′-to-3′ polarity [11, 12]. Because of their unique ring architecture, circRNAs are inherently resistant to exonuclease-mediated degradation and exhibit increased stability compared with their corresponding parental genes [13]. Additionally, circRNAs usually display evolutionary conservation in terms of expression levels, and certain circRNAs have significantly increased expression than corresponding parental genes [14]. In recent years, numerous circRNAs have been discovered to participate in GC genesis and development. Zhang et al. had reported that the circRNA circNRIP1 is wildly expressed in GC to enhance GC cell growth, invasion, and migration [15]. After that, a few circRNAs were reported to be involved in the progression of GC [15], including circMRPS35, circKIAA1244, and circCUL2 as potential GC biomarkers [16–18]. With recent technological breakthroughs in molecular biology, the ability of circRNAs to regulate tumors has been gradually uncovered. It is now extensively accepted that circRNAs are “molecular sponges” that influence microRNAs (miRNAs) functions by complementary binding to the latter [19]. The adsorption capacity of circRNAs to microRNAs is much stronger than that of linear mRNAs and lncRNAs, and thus, the role of circRNAs as endogenous RNAs has been widely concerned. Luo et al. had reported that circCCDC9 sponged miR-6792-3p for inhibiting GC development [20], circACVR2A sponged miR-1290 to regulate GC progression [21], and circ_0043691 sponged miR-873-3p to promote GC progression [22]. These studies supported the hypothesis that circRNAs could be new markers for diagnosing GC and anti-GC therapeutic targets. Bai concluded that 285 dysregulated circular transcripts in LUAD tissues using Gene Ontology (GO) and Kyoto Encyclopedia of Genes and Genomes (KEGG) analysis, and interaction analysis showed that hsa_circ_0002360 was the most significantly overexpressed in LUAD tissues [23]. The data confirmed that circ_0002360 could promote LUAD progression. However, its functions and underlying mechanisms is still unclear in GC.

The article "Circular RNA hsa_circ_0002360 Promotes Proliferation and Invasion and Inhibits Oxidative Stress in Gastric Cancer by Sponging miR-629-3p and Regulating the PDLIM4 Expression" was retracted in 2023. Reasons: unreliable results or conclusions; lack of ethics approval or compliance; concerns about the data; concerns about the peer review.

## 2. Materials and Methods

### 2.1. Microarray Datasets

The present study compared gene levels in GEO-derived GC cases to those in matched healthy tissues. Meanwhile, high-throughput sequencing (HTS) datasets, including GSE103236, GSE79973, GSE33429, GSE22804, and GSE84437, were obtained. The GSE22804 dataset contains 14 normal samples, while the GSE103236 dataset contains 10 GC tumor samples and 9 normal samples. The GSE7997 dataset contains GC and matched healthy samples from 20 cases. GSE33429 dataset includes 27 GC tumor samples. GSE84437 dataset includes 433 GC tumor samples.

### 2.2. Microarray Data Integration and Differentially Expressed Genes (DEGs) Analysis

Possible variables and heterogeneity have frequently been identified as the main variability and bias sources. This work collected datasets from several platforms and treated samples at different times by diverse staff or groups. Consequently, using the R software packages limma and sva, these 4 datasets were integrated by batch normalization to increase sample size (47 cancer along with 33 healthy samples) while avoiding unreliable outcomes. Thereafter, DEGs were identified (*P* < 0.05) between cancer and healthy samples using limma package of R. After integration, genes with abnormal expression levels were preserved in subsequent analyses.

The article "Circular RNA hsa_circ_0002360 Promotes Proliferation and Invasion and Inhibits Oxidative Stress in Gastric Cancer by Sponging miR-629-3p and Regulating the PDLIM4 Expression" was retracted in 2023. Reasons: unreliable results or conclusions; lack of ethics approval or compliance; concerns about the data; concerns about the peer review.

### 2.3. TCGA Data and Differential Expression Analysis

This study also obtained clinical information and gene mRNA expression profiles from the TCGA database (https://portal.gdc.cancer.gov) for 375 GC and 32 matched noncarcinoma samples. To be specific, the data extracted included age, gender, pathological stage, vital status, grade, and TNM stage.  Table 1 presents more detailed patient information. Because all data were obtained from TCGA, there was no need for Ethics Committee approval. Thereafter, DEGs were identified between cancer and healthy samples with limma package of R upon the logFC>1 and *P* < 0.05 thresholds.

### 2.4. WGCNA for the GC-Related Data

Weighted correlation network analysis (WGCNA) was also used in this study to create a weighted gene coexpression correlation network. Meanwhile, “Pearson” correlation coefficients were adopted to determine distances between diverse transcripts. The signless topological overlap matrix (TOM), the minimal module size = 30, and the *β* − power = 9 were utilized to detect coexpressed gene modules and construct the WGCNA network. The significant tumor group-related modules were identified through assessing the relation of coexpression gene modules with tumor or healthy groups. Thereafter, the most significant tumor-related modules with the highest correlation coefficients were chosen for subsequent analysis.

### 2.5. Construction of the GC Model

Survival analysis was completed using qualified datasets (GSE84437, module_bule) with sufficient survival data. Thereafter, genes that predicted overall survival (OS) for GC cases were evaluated by univariate Cox regression. Thereafter, genes with *P* < 0.05 upon univariate Cox regression were selected with glmnet package of R by adopting the least absolute shrinkage and selection operator (Lasso) Cox model. Additionally, those as-selected genes with low lambda were later adopted for constructing the GC prognosis prediction model. Typically, the GC formula was developed by determining selected gene expression weighted by related coefficients. To investigate the relationship of prognostic genes in the GC model with the risk score of OS, the risk score distribution, ROC curve, and scatter plot were adopted.

### 2.6. Function Enrichment Analysis of DEGs

GO offers a framework for depicting gene products' roles in living bodies and identifying typical transcriptome data and biological functions of high-throughput genomes. In general, GO annotations are divided into 3 classes, including biological processes (BPs), molecular functions (MFs), and cellular components (CCs). KEGG analysis can be used to analyze the significant pathways enriched by DEGs, and it may be adopted to interpret gene functions and applied in genome information. Gene functions were analyzed by using the Database for Annotation, Visualization, and Integrated Discovery (DAVID) 6.8 (https://david.ncifcrf.gov). By adopting the related DAVID module, data were converted into biological significance, and datasets were rapidly analyzed at genome level. For revealing whether our selected DEGs were significant for HNSCC development, this study utilized DAVID for GO functional annotation as well as KEGG analysis on DEGs by Venn package, with the significance level set at FDR<0.05.

The article "Circular RNA hsa_circ_0002360 Promotes Proliferation and Invasion and Inhibits Oxidative Stress in Gastric Cancer by Sponging miR-629-3p and Regulating the PDLIM4 Expression" was retracted in 2023. Reasons: unreliable results or conclusions; lack of ethics approval or compliance; concerns about the data; concerns about the peer review.

### 2.7. The Determination of the Biomarkers

Univariate Cox (uni-Cox) regression was conducted to obtain hazard ratios (HRs) (*P* < 0.05). Thereafter, the “survminer” and “survival” packages were employed to detect critical biomarkers. Additionally, randomSurvivalForest was employed to determine a random forest for ranking survival-associated markers in terms of their importance; finally, markers with the relative importance >0.7 were selected. Then, the optimal threshold was applied in the survival analysis, survival curves were drawn using the Kaplan-Meier (KM) approach, and differences were assessed by log-rank test. In addition, this study employed the ggrisk package to draw the scatter plot of biomarker levels as a function of GC survival time. Uni-Cox and multivariate Cox (multi-Cox) regression was subsequently performed using forest plot. Furthermore, prognosis prediction ability of the model was evaluated by receiver operating characteristic (ROC) curve analysis as well as concordance index (c-index) value.

### 2.8. Actinomycin D and RNase R Treatment

DMSO (Sigma-Aldrich, St. Louis, MO, USA) or 2 mg/mL actinomycin D was added to the culture medium to inhibit transcription as the control. Thereafter, total RNA (5 mg) was incubated with/without 3 U/mg RNase R (Epicenter Technologies) for a 30-min period at 37°C, while the RNeasy MinElute Cleaning Kit (QIAGEN, Germany) was later utilized to purity the resultant RNA. Afterwards, total RNA was prepared into cDNA through reverse transcription, and qRT-PCR was conducted to measure hsa_circ_0002360 and GADPH levels.

### 2.9. Dual-Luciferase Reporter Assay

The circular RNA interactome and TargetScan database were adopted for predicting the miR-629-3p binding sites for circ_0002360 or PDLIM4. The Dual-Luciferase Assay System Kit (Promega, Madison, WI, USA) was used to detect dual-fluorescein receptor gene in accordance with specific protocols. After amplification, the mutant (MUT) and wild-type (WT) PDLIM4 3′UTR and hsa_circ_0002360 UTRs were inserted into the luciferase reporter vector pmirGLO (Promega). Thereafter, miR-629-3p mimics were cotransfected into HEK293T cells with luciferase plasmids for a 48-h period. Thereafter, the Dual-Luciferase Reporter Assay System (Promega) was employed to measure luciferase activities, with Renilla luciferase activity serving as a reference for normalizing firefly activity.

The article "Circular RNA hsa_circ_0002360 Promotes Proliferation and Invasion and Inhibits Oxidative Stress in Gastric Cancer by Sponging miR-629-3p and Regulating the PDLIM4 Expression" was retracted in 2023. Reasons: unreliable results or conclusions; lack of ethics approval or compliance; concerns about the data; concerns about the peer review.

### 2.10. RIP Assay

Magna RIP RNA-Binding Protein Immunoprecipitation Kit (Millipore, Billerica, MA, USA) was used for the RIP assay in line with specific protocols. Anti-immunoglobulin G (IgG) and anti-Ago2 antibodies used in the RIP assays were provided by Millipore. qRT-PCR was conducted to measure circRNA and miRNA levels in the collected total RNA.

### 2.11. CircRNA Localization

This study used the Cytoplasmic and Nuclear RNA Purification Kit (Amyjet) to separate and draw cytoplasmic and nuclear RNAs within GC cells in order to determine circRNA localization. Later, circ_002360 expression in cytoplasmic/nuclear RNAs was detected by qRT-PCR, with GAPDH and U5 being the references, separately.

### 2.12. Measurement of Intracellular ROS Levels

The DCFH-DA approach was utilized to measure the relative changes in ROS levels. The cells were incubated for thirty minutes with 10 mmol/L OD DCFH-DA 48 hours after transfection. After three washes, the cells were placed on a fluorescence analyzer (BioTek, USA), and the excitation/emission wavelength was set to 488/525 nm. The results were then analyzed. The values are shown as a percentage of the relative fluorescence of the control group in comparison to the experimental group.

### 2.13. ELISA

Using the appropriate ELISA kits, SOD, CAT, and GSH-PX activities could be measured (Sangon Biotech, Shanghai, China). In a nutshell, the cells were collected before being centrifuged at 1000 g for ten minutes. The instructions were followed, and the supernatant was collected and measured. Gather the supernatant and perform the measurements as directed [24].

### 2.14. Cell Culture as well as Transfection

In this study, human GC cells (NCI-N87, SNU-484, MKN-74, SGC-7901, and AGS) were cultivated together with healthy human gastric epithelial GES-1 cells (Cell Bank, Shanghai, China) in RPMI-1640 medium containing penicillin/streptomycin (Invitrogen, Carlsbad, CA, USA) as well as fetal bovine serum (FBS), followed by incubation with 5% CO_2_ at 37°C. Thereafter, circ_0002360/PDLIM4 overexpression (OE circ_0002360/PDLIM4), shRNA against PDLIM4 (sh PDLIM4), miR-629-3p mimics (miR-629-3p) and inhibitors (miR-629-3p inhibitor), and controls (RiboBio, Guangzhou, China) plasmids were transfected into cells by the use of Lipofectamine 2000 (Thermo Fisher, Waltham, MA, USA). qRT-PCR was conducted to measure transfection efficiency.

The article "Circular RNA hsa_circ_0002360 Promotes Proliferation and Invasion and Inhibits Oxidative Stress in Gastric Cancer by Sponging miR-629-3p and Regulating the PDLIM4 Expression" was retracted in 2023. Reasons: unreliable results or conclusions; lack of ethics approval or compliance; concerns about the data; concerns about the peer review.

### 2.15. qRT-PCR

TRIzol (Invitrogen) was applied to collect total cellular and tissue RNAs, and later the collected RNAs were prepared into cDNA through reverse transcription using PrimeScript RT Kits (Invitrogen). This work utilized the Mx3000P real-time PCR system (Thermo Fisher) for qRT-PCR using SYBR Green SuperMix (Roche, Basel, Switzerland). PCR conditions were shown below, 15 s under 94°C, 10 s under 60°C, and 20 s under 72°C for altogether 40 cycles. Subsequently, 2^-∆∆Ct^ approach was utilized for data analysis, with GAPDH and U6 being the internal references. All primers are listed in Table 2.

### 2.16. Colony Formation Analysis

Cells (2 × 10^4^) were seeded into 6-cm plates and incubated for a 14-day period. Afterwards, methanol was added to fix colonies for a 20-min period (Beyotime, Nanjing, China), followed by 0.1% crystal violet staining (Beyotime), assessment, and count of colonies under the microscope (Olympus, Tokyo, Japan).

### 2.17. Transwell Invasion Assay

Cells (2 × 10^4^) were plated into the Matrigel-coated upper transwell chamber (BD Biosciences) and the RPMI-1640 containing lower chamber. Afterwards, cells were fixed, stained, and observed under the microscope (Olympus).

### 2.18. Western Blotting (WB) Analysis

This work employed RIPA buffer (Beyotime) for extracting total tissue and cell proteins. Thereafter, 12% SDS-PAGE (Beyotime) was performed to separate the extracted proteins, followed by transfer on PVDF membranes (Roche). Then, membranes were blocked using 5% skimmed milk (Beyotime) and incubated with primary antibodies (Abcam, Cambridge, MA, USA) overnight under 4°C, including anti-Ki67 (1 : 1000), anti-MMP9 (1 : 1000), and anti-GAPDH (1 : 5000). Afterwards, the secondary antibody HRP-labeled rabbit IgG (1 : 50,000, Abcam) was employed to further incubate bands. This work adopted enhanced chemiluminescence (ECL, Sangon, Shanghai, China) for protein visualization.

### 2.19. Statistical Analysis

All results were shown in a form of means ± SD. Student's *t*-test was adopted to assess differences in 2 groups, whereas one-way ANOVA was used to assess those among several groups. Significance of difference was analyzed through Spearman correlation. Data were analyzed using SPSS21.0 (IBM, Somers, NY, USA). *p* < 0.05 suggested statistical significance.

## 3. Results

### 3.1. Circ_0002360 Expression Was Increased in GC Cell Lines

Firstly, circ_0002360 expression significantly increased in GC cells in comparison to normal human gastric epithelial cells (Figure 1(a)). Compared with nuclear, cytoplasmic circ_0002360 expression was increased (Figure 1(b)). The results of RNase R assay are that circ_0002360 levels remained largely unchanged after RNase R exposure, whereas linear_0002360 (RUNX1) levels markedly decreased in GC cell lines (Figure 1(c)). As a result, circ_0002360 overexpression plasmids were transfected into GC cells with a lower expression of circ_002360 to upregulate circ_002360 level (Figure 1(d)).

The article "Circular RNA hsa_circ_0002360 Promotes Proliferation and Invasion and Inhibits Oxidative Stress in Gastric Cancer by Sponging miR-629-3p and Regulating the PDLIM4 Expression" was retracted in 2023. Reasons: unreliable results or conclusions; lack of ethics approval or compliance; concerns about the data; concerns about the peer review.

### 3.2. Circ_0002360 Sponged miR-145 for Regulating GC Cell Growth, Migration, and Oxidative Stress

As previously reported, numerous circRNAs are thought to sponge miRNAs; therefore, hsa_circ_00002360's miRNA-binding ability needs to be investigated. A CircInteractome website was utilized to predict target miRNAs of circ_0002360. Among the predicted miRNAs, there were 7 miRNAs (miR-127-5p, miR-758, miR-629, miR-1273, miR-145, miR-933, and miR-585) that were identified according to the score ranked from high to low (Figure 2(a)). miR-629-3p, which was most significantly suppressed following hsa_circ_0002360 overexpression, was adopted in the present work for subsequent analyses (Figure 2(b)). Later, the RIP assay was carried out to pull down RNA transcripts that bound to Ago2 in NCI-H1975 cells. The results of qRT-PCR analysis showed that circ_0002360 and miR-629-3p could be effectively pulled down by anti-Ago2 (Figure 2(c)). Based on luciferase reporter assay, we constructed dual-luciferase reporter vectors containing either the full length of wild-type (WT) circ0002360 or a version where the miR-629-3p-binding site was mutated (MUT) to determine whether miR-629-3p directly targets circ0002360 (Figure 2(d)). The results showed that luciferase activity remarkably decreased within 293T cells after cotransfection of circ_0002360-WT with miR-629-3p mimics (Figure 2(e)). Collectively, the above assays suggest that circ_0002360 can act as miR-629-3p sponges. Next, miR-629-3p mimics was transfected into GC cells to increase its expression (Figure 2(f)). The results of clone formation and transwell assays indicated that the overexpression of circ_0002360 facilitated colony number and invasion in GC cells, while miR-629-3p mimics abolished the above effects (Figure 2(g)). In addition, the enhancing effect of circ_0002360 overexpression on the expression of MMP2 and Ki67 in GC cells was also reversed by miR-629-3p mimics (Figure 2(h)). Next, we found that circ_0002360 overexpression inhibited cellular oxidative stress via reducing ROS level and increasing the levels of SOD, CAT, and GSH-Px (Figure 2(i)–2(l)). However, miR-629-3p mimics abolished the inhibition effects of circ_0002360 overexpression on oxidative stress.

### 3.3. Identification of GC-Related Genes from GEO and TCGA Database

In the present study, we first integrated all samples from GSE103236, GSE22804, GSE33429, and GSE79973 datasets to enlarge the sample size (47 cancer as well as 33 healthy samples; Figure 3(a)). Then, 1874 genes with *P* < 0.05 from the merged dataset were selected (Figure 3(b)). The heatmap of gene expression from TCGA-STAD dataset was shown in Figure 3(c). In TCGA-STAD dataset, a total of 736 DEGs were upregulated or downregulated (Figure 3(d)), then these DEGs were employed to perform GO and KEGG analysis (Figures 3(e) and 3(f)). The 736 DEGs were significantly related to the nuclear division of BP, chromosomal region of CC, and extracellular matrix structural constituent of MF (Sup 1), as well as mostly associated with ECM-receptor interaction and cell cycle pathways (Sup 2).

The article "Circular RNA hsa_circ_0002360 Promotes Proliferation and Invasion and Inhibits Oxidative Stress in Gastric Cancer by Sponging miR-629-3p and Regulating the PDLIM4 Expression" was retracted in 2023. Reasons: unreliable results or conclusions; lack of ethics approval or compliance; concerns about the data; concerns about the peer review.

### 3.4. WGCNA Analysis of Hub Modules for the 736 DEGs

To identify some important GC-related genes, WGCNA was performed. The 80 samples were clustered by Pearson correlation analysis and the average linkage approach, and two outlier samples were excluded from further analyses (Figures 4(a)). Thereafter, we conducted a network topology analysis on diverse soft-thresholding powers to achieve relatively balanced scale independence and WGCNA average connectivity. *β* power was later raised to 9 to construct a scale-free network, with scale-free *R*^2^ reaching 0.86 (Figure 4(b)). Later, this work obtained altogether 5 different modules within the hierarchical clustering tree by means of tree merged-cut dynamics (Figure 4(c)). We discovered 5 different GC modules after merging modules with <25% dissimilarity (Figure 4(d)). In the present study, the modules associated with tumor were considered to be the most important modules. The modules positively associated with GC were the blue (*R* = 0.67; *P* < 0.0001) module. Finally, a total of 83 blue hub genes were screened for further analysis.

### 3.5. Role of mRNA Signature in Predicting OS for Training and Test Cohorts

In the training and testing groups, high-risk cases were associated with increased mortality compared with low-risk cases based on the median risk score (Figures 5(c), 5(d), 5(g), and 5(h)). As suggested by KM analysis, high-risk patients were associated with dismal OS in comparison with low-risk cases from the training group (Figure 5(e)) and testing group (*P* < 0.001; Figure 5(i)). The AUC values of ROC for our constructed 5-mRNA signature were 0.61 and 0.58, respectively, in the training and testing groups (Figures 5(f) and 5(j)), demonstrating that our constructed model well predicted survival of GC.

### 3.6. The Determination of the Key GC-Related Genes

In the merged datasets, differential expression analysis was performed on 27 survival-related risk genes identified by uni-Cox analysis. According to the findings, the 27 genes were found to be downregulated in GC tumor samples (Figure 6(a)). By random forest calculation, we found that MYOC, ABCAB, TMEM100, PDLIM4, PTN, and PDK4 were the key GC-related genes (importance >2) (Figures 6(b) and 6(c)), and their expression was presented in Figure 6(d).

The article "Circular RNA hsa_circ_0002360 Promotes Proliferation and Invasion and Inhibits Oxidative Stress in Gastric Cancer by Sponging miR-629-3p and Regulating the PDLIM4 Expression" was retracted in 2023. Reasons: unreliable results or conclusions; lack of ethics approval or compliance; concerns about the data; concerns about the peer review.

### 3.7. Circ_0002360 Acted as a miR-629-3p Sponge to Affect Cell Proliferation, Invasion, and Oxidative Stress in GC Cells via Promoting PDLIM4 Expression

Firstly, we determined that PDLIM4 was the only one overlapping genes between the six survival-related risk genes and the 5854 target genes of miR-629-3p (Figure 7(a)). The data from GEO and TCGA database verified that GC patients with high expression of PDLIM4 was associated with poor survival in comparison to GC patients with low expression of PDLIM4 (Figures 7(b) and 7(c)). Besides, miR-639-3p mimics suppressed the PDLIM4 level (Figures 7(d) and 7(e)). The results showed that luciferase activity remarkably decreased in 293 T cells subject to cotransfection of PDLIM4-WT with miR-629-3p mimics rather than MUT vector (Figure 7(f)). Then, transfections of OE PDLIM4 and sh PDLIM4 were used to increase PDLIM4 expression and inhibit the expression (Figure 7(i)). Then, circ_0002360 overexpression promoted PDLIM4 expression; meanwhile, the effect was abolished by transfection of miR-629-3p mimics (Figure 7(h)). In addition, the effects of PDLIM4 overexpression on enhancing proliferation and invasion (Figures 7(j)–7(m)) and inhibiting oxidative stress (Figures 7(n)–7(q)) were reversed by miR-629-3p mimics. Circ_0002360 obviously promoted cell proliferation and invasion (Figures 7(r)–7(u)) and suppressed oxidative stress (Figure 7(v)–7(y)), while these effects were eliminated by PDLIM4 knockdown.

## 4. Discussion

CircRNAs can modulate cellular biological behavior to play critical effects on cancer occurrence and development. Because the ring structure is especially stable, circRNAs have been recognized to be the possible targets for tumors diagnosis and prognosis [25]. It reported that circ0002360 expression was upregulated in lung cancer tissues and promoted its progression [23]. Nonetheless, the expression pattern and roles of circ0002360 in GC are still unknown. This work verified that circ0002360 was significantly increased in GC cells in comparison to GES-1 cells, as evidenced by qRT-PCR. According to circRNAs serving as the miRNA sponges in various cancers, the possible target miRNAs of circ0002360 was predicted by adopting the bioinformatics methods. A total of 7 targets were obtained from circular RNA Interactome database. According to qRT-PCR and dual-luciferase assays, circNRIP1 sponged miR-629-3p. In addition, miR-629-3p can promote the progression of breast cancer (BRCA), lung cancer (LC), and head and neck cancer (HNC) [26–29], while it affects the growth, invasion, and migration of cervical cancer (CC) cells [30]. However, the roles and mechanism of miR-629-3p had not been reported in GC. Our results showed that circ0002360 promoted GC cell proliferation and invasion. But miR-629-3p inhibited GC cell proliferation and invasion. However, miR-629-3p mimics abolished the functions of circ0002360 in promoting cell growth and metastasis. It demonstrated that circ0002360 promoted GC progression by sponging miR-629-3p.

The article "Circular RNA hsa_circ_0002360 Promotes Proliferation and Invasion and Inhibits Oxidative Stress in Gastric Cancer by Sponging miR-629-3p and Regulating the PDLIM4 Expression" was retracted in 2023. Reasons: unreliable results or conclusions; lack of ethics approval or compliance; concerns about the data; concerns about the peer review.

Current understanding of the etiology of gastric cancer suggests that oxidative stress plays a role in its progression [31]. Tumor cells have a greater oxidative state, which increases the generation of ROS [32]. In addition, large amounts of reactive oxygen species may boost antioxidant activity in patients with stomach cancer [33]. Past studies have found a rise in CAT activity in patients with tumors [34]. In addition, the activities of GSH, xanthine oxidase, catalase, and copper-zinc superoxide dismutase were considerably elevated in the blood of patients with tumors [35]. Antioxidant enzymes in the mitochondria, such as manganese superoxide dismutase (MnSOD) and glutathione-dependent peroxidase (GPX), are the primary mitochondrial defense system against oxidative stress [36]. Therefore, inhibition of the antioxidant system is therefore a possibility for cancer treatment. In this study, when vectors expressing circ0002360 were transfected into cells, SOD, CAT, and GSH-Px activities rose, while ROS levels dropped. On the other hand, the transfection of miR-629-3p mimics had the opposite effect. Furthermore, miR-629-3p mimics abolished the inhibition of oxidative stress caused by circ0002360 overexpression. Inducing ROS generation to disable the antioxidant defense system has been reported as a novel technique for cancer therapy [37]. Thus, inhibiting circ0002360 decreased gastric cancer cell proliferation and invasion while also increasing the inhibition effects of cell proliferation by promoting ROS generation and decreasing antioxidant activity. This process is inextricably linked to the expression of miR-629-3p.

To determine the target gene of miR-629-3p, we download the GC-related expression profile data from GEO and TCGA database to determine differential expressed genes. Previous studies usually used some target gene prediction websites, such as TargetScan, to screen out target genes of miRNAs [38, 39]. However, we first used WGCNA and uni-Cox analysis to construct a risk model for prognosis prediction. Next, randomForest analysis identify key survival-related risk signatures. Finally, Venn analysis determined a target gene of miR-629-3p from TargetScan database and risk signatures termed PDLIM4. Our results are obtained from multiple databases with different analyses. Therefore, it had a higher degree of confidence.

The article "Circular RNA hsa_circ_0002360 Promotes Proliferation and Invasion and Inhibits Oxidative Stress in Gastric Cancer by Sponging miR-629-3p and Regulating the PDLIM4 Expression" was retracted in 2023. Reasons: unreliable results or conclusions; lack of ethics approval or compliance; concerns about the data; concerns about the peer review.

PDLIM4 (reversion-induced LIM domain) is a tumor suppressor gene located at 31.1 on the long arm of chromosome 5 and can encode one adapter protein, which belongs to ALP/Enigma family and has high conservation degree [40]. Because PDLIM4 has domains (LIM and PDZ), PDLIM4 can be the scaffold that interacts with membrane receptors and cytoplasmic signal molecules, as well as actin-related proteins [41]. PDLIM4 is identified to be a tumor suppressor [42] and shows abnormal expression in different cancer types. For BRCA, the abnormal expression of PDLIM4 is closed related to tumor clinical features, like cell ploidy, tumor size, SPF (S-phase fraction), and differentiation status [43]. Besides, PDLIM4 regulates the expression of proto-oncogene to promote cell proliferation, invasion, and active angiogenesis pathways [44, 45]. Based on cell experiment in this work, miR-629-3p target PDLIM4 and served as the tumor suppressor in GC. It showed that miR-629-3p inhibited the progression GC. Next, we used rescue experiments to verify the relation of circ0002360, miR-629-3p, and PDLIM4 in GC cells. The results showed that miR-629-3p mimics could reverse the effects of circ0002360 and PDLIM4 overexpression on GC cell phenotypes, and PDLIM4 knockdown could abolish the regulated effects of circ0002360 overexpression on GC cell proliferation, invasion, and oxidative stress. Therefore, circ0002360 sponged miR-629-3p to exert its function in GC progression. Besides, circ0002360 positively regulated PDLIM4 to promote cell proliferation and invasion and inhibit oxidative stress. CircRNAs could sponge several miRNAs to regulate cell proliferation and might be the oncogene in several cancer types, which sponged diverse miRNAs (concurrently or not) because of the certain tissues and cells implicated. In this work, circ0002360 exerted its effects through sponging miR-629-3p in GC cells, at least partly.

### 4.1. Limitation

CircRNAs-medicated effects in cell proliferation, invasion, and so on dependent on the abundance of miRNA and the number of miRNA-binding site. Consequently, the above observations might be change because of the different circ0002360, miRNA targets, and miRNAs expression levels within diverse cells. Therefore, more studies are needed to explore the mechanism of circ0002360 in the action mode in diverse malignancies. Furthermore, this study merely confirmed the role and molecular mechanism of the circ0002360/miR-629-3p/PDLIM4 axis in gastric cancer at the cellular level, with no clinical or animal involvement. Furthermore, bioinformatics approaches were used to examine the stomach cancer-related expression profile data in public databases (TCGA and GEO database), and no comparable clinical cases were obtained for examination, resulting in a lack of clinical guidance. As a result, in the follow-up investigation, we will collect clinical samples and conduct relevant animal studies to clarify the roles and molecular mechanisms of the circ0002360/miR-629-3p/PDLIM4 axis in gastric cancer.

The article "Circular RNA hsa_circ_0002360 Promotes Proliferation and Invasion and Inhibits Oxidative Stress in Gastric Cancer by Sponging miR-629-3p and Regulating the PDLIM4 Expression" was retracted in 2023. Reasons: unreliable results or conclusions; lack of ethics approval or compliance; concerns about the data; concerns about the peer review.

In conclusion, this work suggests the upregulation of circ0002360 in GC cells accelerates GC cell proliferation, invasion, and inhibits oxidative stress through sponging miR-629-3p to increase PDLIM4 expression. This work offers further evidence supporting the roles of circRNAs in sponging miRNAs, which indicates that circ0002360 is the possible marker to predict GC prognosis and the anti-GC therapeutic target.

## Figures and Tables

**Figure 1:** Circ_0002360 was elevated in GC cell lines. (a) The expression of circ_0002360 in cells was detected by qRT-PCR. (b) qRT-PCR analysis of hsa_circ_0002360, GAPDH, and U6 in the cytoplasm and nucleus in LUAD cells. (c) The stability of circ_0002360 by RNase R assay. (d) QRT-PCR analysis of hsa_circ_0002360 expression in cells transfection with circ0002360 overexpression. Data in the represent the mean values ± SD from three biological replicates (*n* = 3). ∗*P* < 0.05.

**Figure 2:** Circ_0002360 sponged miR-145. (a) A schematic illustration demonstrating the putative binding sites of the miRNAs associated with hsa_circ_0002360. (b) qRT-PCR data show expressions of the candidate miRNAs after hsa_circ_0002360 overexpression in cells. (c) qRT-PCR for the expression of hsa_circ_0002360 and miR-145 in cells after pulling down of Ago2 by RIP assay. (d) A schematic of wild-type (WT) and mutant (MUT) hsa_circ_0025202 luciferase reporter vectors. (e) The luciferase activity of WT hsa_circ_0002360 3′ UTR or mutant hsa_circ_0002360 30'UTR after transfection with miR-629-3p mimics in cells. (f) The transfection efficiency of miR-145 mimics in cells were evaluated by qRT-PCR. (g) Colony numbers was detected using colony formation assay, and cell invasion was measured with transwell assay. (h) Ki67 and MMP9 expression in cells was detected by western blotting. (i) The production of ROS was measured by DCFH-DA method. (j–l) The activity of SOD, CAT, and GSH-Px was measured by ELISA. Data in (b, c, e, f, g, h, i, j, k, and l) represent the mean values ± SD from three biological replicates (*n* = 3). ∗*P* < 0.05.

The article "Circular RNA hsa_circ_0002360 Promotes Proliferation and Invasion and Inhibits Oxidative Stress in Gastric Cancer by Sponging miR-629-3p and Regulating the PDLIM4 Expression" was retracted in 2023. Reasons: unreliable results or conclusions; lack of ethics approval or compliance; concerns about the data; concerns about the peer review.

**Figure 3:** Identification of GC-related genes from GEO and TCGA database. (a) Principal component analysis (PCA) of analysis of integrated datasets from GSE103236, GSE22804, GSE33429, and GSE79973 datasets. (b) Heatmap of GEO-derived DEGs with *P* value <0.05. (c) Heatmap of TCGA-derived DEGs with logFC>1 and *P* value <0.05. (d) Heatmap of TCGA- and GEO-derived DEGs. GO (e) annotation and KEGG (f) pathways analysis of the DEGs.

**Figure 4:** WGCNA analysis of hub Modules for the 736 DEGs (a) Clustering dendrogram of 80 samples and excluding two outlier sample. (b) Analysis of the scale-free fit index for various soft-thresholding powers (*β*) and analysis of the mean connectivity for various soft-thresholding powers. (c) The dendrogram of all genes is clustered based on a dissimilarity measure (1-TOM). (d) The heatmap shows the correlation among MEs, normal, and tumor. Red represents a positive correlation between modules and clinical characteristics, and blue represents a negative correlation between modules and clinical characteristics.

**Figure 5:** Prediction of the mRNA signature for over survival in the train group and test group. (a) Venn analysis of overlapping genes between GSE84437 dataset and blue module. (b) Uni-Cox analysis of the 83 overlapping genes. (c, g) The curve of risk score in training group and testing group; (d, h) survival status by ggrisk in training group and testing group. (e, i) Survival analysis in training group and testing group. (f, j) ROC cure analysis in training group and testing group.

**Figure 6:** The Determination of the Key GC-related genes (a) Heatmap of 27 survival-related risk genes expression in the merged datasets. (b) the tree of randomForest; (c) variable relative importance of randomForest. (d) Heatmap of 6 survival-related risk signatures expression in the merged datasets.

**Figure 7:** Circ_0002360 acted as a miR-629-3p sponge to affect cell proliferation, invasion, and oxidative stress in GC cells via promoting PDLIM4 expression (a) Venn analysis of overlapping genes between the risk signatures and target genes of miR-629-3p. The survival status between PDLIM4 high expression group and the low expression group in GEO database (b) and TCGA database (c). (d) The transfection efficiency of PDLIM4 overexpression in cells were evaluated by western blotting and qRT-PCR assay. (f) A schematic of wild-type (WT) and mutant (MUT) PDLIM4 luciferase reporter vectors. (g) The luciferase activity of WT PDLIM4 3′ UTR or mutant hsa_circ_0002360 30′UTR after transfection with miR-629-3p mimics in cells. The PDLIM4 expression (h), cell proliferation (j, l), invasion (k, m), ROS (n), and the levels of SOD, CAT, and GSH-Px (o–q) in cells transfection with circ0002360 overexpression and miR-629-3p mimics were evaluated by western blotting and qRT-PCR assay, colony formation assay, and transwell assay. Cell proliferation (r, t), invasion (s, u), ROS (v), and the levels of SOD, CAT, and GSH-Px (w–y) in cells transfection with circ0002360 overexpression and PDLIM4 knockdown were evaluated by colony formation assay and transwell assay. Data in (d, e, and g–y) represent the mean values ± SD from three biological replicates (*n* = 3). ∗*P* < 0.05 and #*P* < 0.05.

The article "Circular RNA hsa_circ_0002360 Promotes Proliferation and Invasion and Inhibits Oxidative Stress in Gastric Cancer by Sponging miR-629-3p and Regulating the PDLIM4 Expression" was retracted in 2023. Reasons: unreliable results or conclusions; lack of ethics approval or compliance; concerns about the data; concerns about the peer review.

**Table 1:** Characteristics of patients with GC from TCGA database.

Characteristics	Variable	Patients (375)	Percentages (%)
Age	<65 years	155	41.33
	≥65 years	216	57.60
	Unknown	4	1.07
Gender	Male	241	64.27
	Female	134	35.73
Grade	G1	10	2.67
	G2	137	36.53
	G3	219	58.40
	GX	9	2.40
Pathological stage	I	53	14.13
	II	111	29.60
	III	150	40.00
	IV	38	10.13
	Unknown	23	6.14
T classification	T1	19	5.07
	T2	80	21.33
	T3	168	44.80
	T4	100	26.67
	TX	8	2.13
N classification	N0	111	29.60
	N1	97	25.87
	N2	75	20.00
	N3	74	19.73
	NX	16	4.27
	Unknown	2	0.53
M classification	M0	330	88.00
	M1	25	6.67
	MX	20	5.33
Vital status	Alive	244	65.07
	Death	131	34.93

GC: gastric cancer. Data are presented as number (%).

**Table 2:** The sequences of the primers.

Gene	Forward (5′-3′)	Reverse (5′-3′)
circRNA_0002360	AGAAACTAAGGCACAGCTAAACA	GGGCGAAAAATGTCCAG
miR-145	AGTCCCTGCAGATATAGCTACAA	AGACGTCAAGGCGGTAGGTAGTT
miR-127-5p	ATGTGTCCGTGTCCGACGTGAAA	CTGTGTCATGTGTCAATGTCCT
miR-758	TGTGTCCACCATGACGATCGTGTC	CTGTGTAAACGTAACGACGACT
miR-629	GCTGTGTAACGCTTGTGAAAGTAA	CGATGTGACGCGCTGGGCAA
miR-1273	AACGCTAACGTGCCATGTGTAA	CCCCATGTAACGTGCAAATGTGT
miR-933	TTGCTAACGCTAAGCTGCAATGG	AACGCTGTAGTGTAGAGATGATA
miR-585	CCGCTAGTGTAACGTGAAACGCCA	CCATGTGAATGTAGTAGTAACC
PDLIM4	GCAACGCATGTCTGTGTAACA	AATGTGTAAGTGTAAACCATGCG
U6	TTCGGCACGCAGTTGACTCGC	ACGAAACCGTCTTGCTAAGG
GAPDH	TTAAATTGCCCCCAGCCAACTT	ACACACAGGCGGCACCATA

## Data Availability

Data will be available upon reasonable request.

## Supplementary Materials

Supplementary Materials Supplementary Table 1.: GO analysis. Supplementary Table 2: KEGG pathway.
